# Anti-wrinkle effects of fermented and non-fermented *Cyclopia intermedia* in hairless mice

**DOI:** 10.1186/1472-6882-14-424

**Published:** 2014-10-29

**Authors:** A-Rang Im, Jae Hyoung Song, Mi Young Lee, Sung Hum Yeon, Key An Um, Sungwook Chae

**Affiliations:** KM-Based Herbal Drug Development Group, Korea Institute of Oriental Medicine, 1672 Yuseongdae-ro, Yuseong-gu, Daejeon 305-811 Korea; Research Center, Huons Co. Ltd, 55 Hanyangdaehak-ro, Sangrok-gu, Ansan, Gyeonggi-do 426-791 Korea

**Keywords:** Anti-wrinkle, *Cyclopia intermedia*, Honeybush, Fermented honeybush, Photoaging

## Abstract

**Background:**

The fermented leaves and stems of *Cyclopia intermedia* are used to brew honeybush tea, an herbal tea indigenous to South Africa with reported anti-wrinkle effects. Wrinkle formation caused by photoaging clearly involves changes in extracellular matrix components and mechanical properties of the skin.

**Methods:**

The inhibitory effects of honeybush extract and fermented honeybush on wrinkle formation were determined by analyzing skin replicas, histologically examining epidermal thickness, and identifying damage to collagen fibers.

**Results:**

Honeybush extract and fermented honeybush reduced the length and depth of skin winkles caused by UV irradiation and inhibited thickening of the epidermal layer, in addition to suppressing collagen tissue breakdown reactions, indicating its potential use as a skin wrinkle prevention agent.

**Conclusions:**

This *in vivo* study demonstrates that honeybush produces significant anti-wrinkle effects and is therefore of interest in anti-aging skin care products.

## Background

The most representative symptom of skin aging is wrinkling [1]. Skin aging is influenced by inherited intrinsic factors and by extrinsic or environmental factors, such as chronic UV radiation. Skin photoaging by UVB radiation is clinically and histologically distinct from the natural aging process of the skin, and is characterized by wrinkles, uneven pigmentation, brown spots, laxity, and a leathery appearance [2]. The UVB are mostly responsible for skin changes such as wrinkle formation, epidermal thickening, degradation of matrix macromolecules, vascularization, and immunosuppression. However, UVA is partly absorbed and has lower efficiency in skin damage like erythema [3–5].

To reduce skin wrinkles and other skin diseases, various chemicals like retinol and its derivatives are used in cosmetics and medicines [6]. However, these materials have the disadvantages of high price and chemical instability, which reduces their practicality. Therefore, the development of safer and more effective treatments for the alleviation of skin wrinkles has been an important focus of study in the medical, food, and cosmetic industries. Traditionally used herbal medicines derived from plants represent a productive base from which to search for such bioactive compounds. Furthermore, fermentation has been shown to improve the therapeutic effects of some herbal medicines [7, 8].

The fermented leaves and stems of *Cyclopia intermedia* are used to brew honeybush tea, an herbal tea indigenous to South Africa [9]. Honeybush is a flowering plant belonging to the family Fabaceae, which is found only in a narrow area of mountain ridges in the cape region of South Africa, and shows great similarity to rooibos [10]. Honeybush is used traditionally for medicinal purposes, is rich in polyphenols, and with rooibos is a rare source of the dietary dihydrochalcones, aspalathin and nothofagin [11]. Antioxidant activity of honeybush extracts has been confirmed by *in vitro* and *in vivo* test [12, 13]. In vitro antioxidant activity of water extracts have antioxidant activity as compared to the other teas.

In previous research, honeybush extracts protected the skin via modulation of induced-oxidative damage, inflammation and cell proliferation [14]. And also, honeybush inhibited tomour promotion that modulated biological events involved during 12-*O*-tetradecanoylphorbol-13-acetate (TPA) -induced tomour promotion in mouse skin [15]. This would imply that honeybush can protect skin damage against UVB-induced mouse skin. Most recently, we have shown that oral feeding of *Mangifera indica* L. to mice enhanced the skin aging against UVB-induced hairless mice model [16]. And also, mangiferin isolated from *Anemarrhena asphodeloids* had an inhibition effect of UVB-induced wrinkle formation and MMP-9 expression [17]. But whether and how honeybush improves anti-wrinkle effects are unknown which was impetus of our research. In this study, we investigated the anti-wrinkle effects of honeybush extract and fermented honeybush in a hairless mice model. More specifically, we examined the effect of honeybush extract and fermented honeybush on UVB-induced photoaging in the skin of hairless mice by evaluating various parameters of photoaging.

## Methods

### Materials

Honeybush was purchased from Renewallife [http://www.renewallife.com, Korea, a voucher specimen (KIOM-HB 2010)] in a herbarium in which the temperature was maintained at 5.5 ± 0.3°C and the humidity was maintained at 50 ± 5%. HR-1 hairless male mice (6 weeks of age) were purchased from Japan SLC, Inc. (Shizuoka, Japan). UVB radiation was administered using a UVM-225D Mineralight UV Display Lamp (UVP, Phoenix, AZ, USA). Replicas of mouse dorsal skin were obtained using a Repliflo Cartridge Kit (CuDerm Corp., Dallas, TX, USA).

### Preparation of honeybush extract and fermented honeybush

The dried plant materials (25 g) were extracted with distilled water (220 mL) two times under reflux for 1 hr and were then filtered through filter paper. The filtrate was evaporated to dryness in vacuo to yield a red powder (4.3 g). To prepare fermented honeybush, 1 mL of lactic acid bacteria (*Streptococcus thermophilus*, 3 × 10^5^ CFU/mL) cultured in MRS (de Man, Rogosa, & Sharpe) medium was inoculated in 100 mL of milk with 3 g of sugar and the honeybush extract (5%, w/v), and the mixture was fermented in a 37°C incubator for 1 day.

### Experimental animals and oral administration

All experimental protocols were approved by the Korea Institute of Oriental Medicine Institutional Animal Care and Use Committee (10-094). HR-1 hairless male mice (6 weeks of age) were purchased from Japan SLC, Inc. (Shizuoka, Japan) and allowed to habituate for 1 week prior to the study. The animals were housed in climate-controlled quarters (24°C at 50% humidity) with 12 h light/dark cycles and had free access to food and water. The mice were divided into control (n =5), UVB-treated vehicle (n =5), UVB-treated honeybush (n =5), and UVB-treated fermented honeybush (n =5) groups. Mice from the honeybush extract group were orally administered 0.1 mL of water containing 100 mg/kg of honeybush each day prior to UVB irradiation. The fermented honeybush-treated group mice were fed 0.1 mL of the fermented honeybush mixture. Drinking water was supplied to animals in the vehicle group, and the unexposed control group was not treated with any material.

### UVB irradiation

UVB irradiation was performed using a UVM-225D Mineralight UV Display Lamps (UVP, Phoenix, AZ, USA) emitting at a wavelength of 302 nm. UV strength was measured using an HD2102-2 UV meter (Delta OHM, Padova, Italy). UVB radiation was applied to the backs of the mice three times per week for 12 weeks. The amount of irradiation was progressively increased from 60 mJ/cm^2^ per exposure at week 1 (1 minimal erythematous dose =60 mJ/cm^2^) to 90 mJ/cm^2^ at week 7.

### Generation of replicas and image analysis

Replicas of mouse dorsal skin were obtained using the Repliflo Cartridge Kit (CuDerm Corp., U.S.A.). A photograph of the dorsal skin was taken before the animals were sacrificed. The impression replicas were set on a horizontal sample stand and wrinkle shadows were produced by illumination with a fixed-intensity light at a 35° angle using an optical light source. Black and white images were recorded with a CCD camera and analyzed by Skin-Visiometer VL 650 software (Courage & Khazaka, Cologne, Germany). The parameters used in the assessment of skin wrinkles were the average length and average depth of wrinkles.

### Histological examination

Dorsal skin was fixed in 10% neutral buffered formalin, embedded in paraffin, and sectioned at 5 μm. Sections were stained with hematoxylin and eosin (H&E) and Masson's trichrome for collagen fiber analysis. The thickness of the epidermis was measured under light microscopy with an eyepiece micrometer (Olympus, Japan).

### Statistical analysis

All measurements were made in triplicate and all data are presented as mean ± standard error of the mean (SEM). The results were subjected to analysis of variance (ANOVA) using Tukey’s multiple comparison test to analyze differences, and *p* <0.05 was considered to be significant.

## Results

### Evaluation of wrinkle alleviation effects by replica images

As shown in Figure 1, thick and deep wrinkles formed along with fine wrinkles in the UVB-irradiated group, compared with the control group. In the honeybush extract-treated group and the fermented honeybush-treated group, the thickness and depth of wrinkles caused by UVB irradiation was alleviated (Figure 1). Therefore, it was confirmed that the honeybush extract and fermented honeybush mixture alleviated skin wrinkles caused by UVB irradiation.

**Figure 1:** **Effects of honeybush extract and fermented honeybush on UVB-induced wrinkle formation.** Analysis of wrinkles was performed using skin replicas taken from the dorsal skin. Analysis of the replica images was performed using Skin-Visiometer software. HB = honeybush extract, STC HB = fermented honeybush.

### Mean length and depth of wrinkles by replica analysis

To quantitatively analyze the wrinkle alleviation effect of the honeybush extract and fermented honeybush, the length and depth of wrinkles were investigated. As shown in Figure 2, the mean length and depth of wrinkles were increased in the UVB-irradiated group compared with the wrinkles of the control group. The length of wrinkles in the honeybush extract-treated group was decreased 8.9% compared to those of the UVB-irradiated group. The length of wrinkles in the fermented honeybush-treated group was decreased 28% compared to the UVB-irradiated group. As shown in Figure 2B, the depth of wrinkles in the fermented honeybush treated group was decreased 17% compared to those of the UVB-irradiated group, which a statistically significant difference (*p* <0.05).

**Figure 2:** **Analysis of the replica images was performed using Skin-Visiometer software for the determination of (A) mean length, and (B) depth of wrinkles.** Data are reported as relative percentages of the UVB group measurements. * *p* <0.05; HB = honeybush extract, STC HB = fermented honeybush.

### Evaluation of anti-wrinkle effects by histological staining in UVB-irradiated hairless mice

To confirm the wrinkle alleviation effect of the honeybush extract and fermented honeybush, skin tissue samples were taken from the hairless mice, followed by histological staining. Skin tissue samples were taken from each hairless mouse and fixed in 10% neutral formalin solution. The fixed tissue samples were washed, dehydrated, cleaned, infiltrated, and embedded in paraffin. The paraffin block was sliced into 4-μm-thick sections that were subjected to hematoxylin and eosin (H&E) staining and Masson's trichrome staining. As shown in Figure 3A, H&E staining confirmed that the thickness of the stratum corneum was significantly increased in the UVB-irradiated group compared to the control group, and the epidermal thickness was increased. However, the stratum corneum thickness was decreased in the honeybush extract-treated group and the fermented honeybush-treated group compared to the UVB-irradiated group, and the epidermal thickness was reduced (Figure 3A).

**Figure 3:** **Effects of honeybush extract and fermented honeybush treatment on UVB-induced skin thickening in hairless mice. (A)** Hematoxylin and eosin staining of UVB-irradiated hairless mouse skin. **(B)** Epidermal thickness of dorsal skin. Original magnification was 200×. Data are reported as relative percentages of the UVB group measurements. * *p* <0.05; HB = honeybush extracts, STC HB = fermented honeybush.

To measure the anti-wrinkle effects of the honeybush extract and fermented honeybush, changes in epidermal thickness were investigated by measuring the distance from the keratin layer to the epidermal basement membrane in the tissue stained with H&E using a ruler-equipped microscope. The significance of the differences in results from the control group and the experimental groups was obtained. As shown in Figure 3B, epidermal thickness was increased in the UVB-irradiated group compared to that of the control group. However, the epidermal thickness in the honeybush extract-treated and fermented honeybush-treated group was reduced 40% and 56%, respectively, compared to the UVB-irradiated group. The anti-wrinkle effect of the fermented honeybush, as indicated by epidermal thickness, was greater than that of the non-fermented honeybush extract (*p* <0.05). Therefore, the honeybush extract and fermented honeybush significantly reduced epidermal thickness, suggesting that they are effective anti-wrinkle agents.

### Collagen staining

As shown in Figure 4, Masson's trichrome staining showed a regular distribution pattern of collagen in the dermal layer. Collagen fibers were increased in the honeybush extract-treated group and the fermented honeybush-treated group compared to the UVB-irradiated group (Figure 4). More collagen fibers were observed in the fermented honeybush-treated group than in the honeybush extract-treated group. These results confirmed that the honeybush extract and fermented honeybush alleviated skin wrinkles caused by UVB irradiation, and the fermented honeybush was more effective than the honeybush extract.

**Figure 4:** **Protective effects of honeybush extract and fermented honeybush on collagen fibers exposed to UVB radiation.** Histological observation of hairless mouse skin was performed using Masson’s trichrome stain. Collagen fibers were stained in blue and pictures were taken at a magnification of 200×. HB = honeybush extract, STC HB = fermented honeybush.

## Discussion

Many antioxidants and anti-photoaging compounds that effectively inhibit skin photodamage are available [18]. A number of experimental studies have confirmed the protective effects of antioxidants against acute and chronic skin photodamage [19]. In this study, we used lactic acid bacteria that are widely used in food fermentation. Fermentation has been shown to improve the therapeutic effect of some herbal medicines, and one of the commonly known functional properties such as antioxidant was widely been studied and discussed [20, 21]. Therapeutic enhancement is reported to relate with the changes in secondary metabolite profiles during fermentation and the mechanisms that affect biological activity are varied [22]. To the best of our knowledge, there is no report on the comparison of anti-wrinkle efficacy according to bioconversion of honeybush extract, in this study, we used lactic acid bacteria that are widely used in food fermentation. The main compounds of the *Cyclopia* plants are polyphenols contains xanthones, flavones, isoflavones, flavanones and coumestans [23]. Research showed that water extracts from both fermented and non-fermented herb of *Cyclopia* plants have considerable antioxidant potential and exhibit antimutagenic properties in vitro, ex vivo and in vivo [9]. Further investigation is needed to identify the precise mechanisms for anti-wrinkle activity based on fermentation.

Skin aging is a multifaceted biological process that is characterized by the appearance of wrinkles, pigmentation irregularities, and loss of firmness, and to which UV light and free radicals make substantial contributions [24]. The skin is the biological tissue most susceptible to solar UV radiation, which is absorbed by various chromophores in the skin, such as melanin, DNA, RNA, proteins, lipids, and water, as well as aromatic amino acids, such as tyrosine [25].

Extrinsic aging refers to components mediated by environmental factors, of which UVB exposure is the most significant [26]. Skin UV radiation exposure causes oxidative stress that leads to inflammatory reactions such as acute erythema and chronic damage [18]. UV radiation also accelerates damage to the epidermis and dermis, resulting in the appearance of wrinkles [27]. Wrinkle formation occurs because of the accumulation of skin damage such as matrix destruction and skin inflammation [28]. In this study, it was confirmed that honeybush extract and fermented honeybush alleviated skin wrinkles caused by UVB irradiation.

The mechanical and elastic properties of the skin that are associated with skin wrinkling are related to the histomorphology of the epidermis [29]. Photoaged skin has a peculiar appearance, with deep wrinkles that are not erased by stretching, pigmentary alterations that include areas of hyper- and hypopigmentation, and a variety of neoformations [30]. Photodamaged skin also shows variable epidermal thickness, decreased and fragmented collagen, increased degradation by matrix metalloproteinases, inflammatory infiltrates, and vessel ectasia [27]. In this study, the effects of UVB irradiation on the stratum corneum were alleviated in the honeybush extract-treated group and the fermented honeybush-treated group, and the epidermal thickness was also reduced. Interestingly, the fermented honeybush was more effective than the honeybush extract. The fermentation group without honeybush had no inhibitory effect on wrinkles in terms of mean length, mean depth, and epidermis thickness (data not shown) as compared to UVB irradiated group.

A large number of commercial anti-wrinkle and anti-aging compounds are available to consumers for rejuvenation of facial skin damaged by age or solar radiation. Anti-wrinkle agents such as retinoic acid, niacinamide, and vitamins have been tested clinically, and laboratory experiments have been conducted in animal models [31–33].

## Conclusions

These results show that oral administration of fermented and non-fermented honeybush prevent UVB-induced wrinkle formation *in vivo*, and that changes in the morphorogical properties of the skin produced by honeybush treatment are due to changes in the epidermis. This *in vivo* study demonstrates that fermented and non-fermented honeybush produce significant anti-wrinkle effects and is therefore of interest in anti-aging skin care products.
